RETRACTED

# The amelioration of alcohol-induced liver and intestinal barrier injury by *Lactobacillus rhamnosus* Gorbach-Goldin (LGG) is dependent on Interleukin 22 (IL-22) expression

**DOI:** 10.1080/21655979.2022.2070998

**Published:** 2022-05-21

**Authors:** Yuli Ge, Huiling Sun, Lanman Xu, Weiping Zhang, Jiaojian Lv, Yongping Chen

**Affiliations:** a Department of Infectious Diseases and Liver Diseases, Lishui People’s Hospital, Lishui, China; b Department of Infectious Diseases and Liver Diseases, Ningbo Medical Centre Lihuili Hospital, Affiliated Lihuili Hospital of Ningbo University, Ningbo Institute of Innovation for Combined Medicine and Engineering, Ningbo, China; c Intervention Therapy Department, Lishui People’s Hospital, Lishui, China; d Department of Infectious Diseases, The First Affiliated Hospital of Wenzhou Medical University, Zhejiang Provincial Key Laboratory for Accurate Diagnosis and Treatment of Chronic Liver Diseases, Wenzhou, China

**Keywords:** Alcoholic liver disease, IL-22 signaling pathway, intestinal barrier injury, LGG, liver function

## Abstract

Alcoholic liver disease (ALD) is a common clinical liver injury disease. *Lactobacillus rhamnosus* Gorbach-Goldin (LGG) has been revealed to alleviate alcohol-induced intestinal barrier and liver injury. However, the underlying mechanism of LGG treatment for ALD remains unclear. To clarify this aspect, a chronic plus binge ALD model was constructed using C57BL/6 mice in line with a chronic alcohol binge feeding protocol. Interleukin 22 (IL-22) level was determined by quantitative real-time polymerase-chain reaction and enzyme-linked immunosorbent assays. Effects of LGG in model or IL-22 knockdown in LGG-treated model on the liver injury and steatosis status, as well as intestinal barrier function were assessed by hematoxylin eosin (HE) staining. Levels of alanine aminotransferase (ALT), triglyceride (TG), and aspartate aminotransferase (AST) in serum were measured by the corresponding kit. Western blot analysis was conducted to detect protein expressions of intestinal tight junction protein 1 (ZO-1) and Claudin-1. Concretely, LGG elevated IL-22 level in liver tissues and serum, while inhibiting ALT, TG, and AST levels in alcohol-exposed mice. Moreover, LGG alleviated liver injury, steatosis, and intestinal barrier injury caused by alcohol, and enhanced ZO-1 and Claudin-1 expressions. Furthermore, IL-22 knockdown increased ALT, TG, and AST levels in serum, and aggravated liver injury, steatosis, and intestinal barrier injury. ZO-1 and Claudin-1 levels were downregulated by IL-22 silencing. Importantly, downregulation of IL-22 reversed the effect of LGG on the liver and intestinal barrier injury. To conclude, LGG protects against chronic alcohol-induced intestinal and liver injury via regulating the intestinal IL-22 signaling pathway.

RETRACTED

## Highlights

- LGG elevated the level of IL-22 in alcohol-exposed mice.
- LGG protected against alcohol-induced liver damage and steatosis, as well as intestinal barrier injury.
- The intestinal IL-22 signaling pathway participated 57 in the hepatoprotective activity of LGG.

## Introduction

Excessive alcohol consumption could lead to several problems, seriously affecting public health in the world [1,2]. One of the cases is alcoholic liver disease (ALD), which is also the main cause of chronic liver diseases globally, could bring about extensive liver damage, including simple fatty liver, alcoholic steatohepatitis, liver fibrosis, cirrhosis, and even hepatocellular carcinoma [3–5]. ALD also exhibits an extremely complicated pathogenesis, mainly containing inflammatory immune response to injury, ethanol-mediated liver injury, and microbiome and intestinal permeability changes [6,7]. Scientists have long sought a safe and effective way to treat and prevent ALD, and despite remarkable progress, complete control toward ALD remains elusive. Fortunately, new pathophysiology-based therapies, such as interleukin 22 (IL-22) and anakinra, have shed light on the treatment of ALD [8]. Previous studies have revealed that IL-22 treatment has antisteatotic, antiapoptotic, antioxidant, proliferative, and antimicrobial effects, demonstrating that it may be a potential option for ameliorating ALD [9]. However, there is still a lack of in-depth investigation on the potential mechanism of its action.

Probiotics have good antioxidant activity and the ability to improve intestinal barrier function [10]. In nearly a decade, researchers have begun to take probiotics as a new way for the prevention and treatment of ALD, especially for *Lactobacillus rhamnosus* Gorbach-Goldin (LGG) [11,12]. LGG is a Gram-positive bacterium that plays an important role in lipid modulation, immunoregulation, and gene expression in diseases, such as ALD, nonalcoholic-liver disease, and inflammatory bowel disease [13]. Wang et al. reported that LGG treatment ameliorates alcohol-induced liver injury, promotes intestinal integrity, and enhances intestinal hypoxia-inducible factor [14]. Moreover, Bruch-Bertani et al. found that LGG exerts a hepatoprotective effect on an alcoholic liver disease model in Zebrafish by regulating gut permeability and inflammasomes [15]. Also, LGG treatment could reduce alcohol-induced hepatic inflammation [16]. Although numerous studies have suggested that supplementation with LGG can effectively ameliorate or prevent alcohol-induced liver injury, the mechanism of the beneficial action has not been well defined.

RETRACTED

Here, we hypothesized that LGG may effectively alleviate alcohol-induced liver injury via modulating the IL-22 signaling pathway. Wild-type mouse model of chronic plus binge ALD was established to explore the effect of LGG on the expression level of IL-22, liver injury, and intestinal barrier. Besides, we managed to fathom out whether LGG generates protective effects on liver injury and intestinal barrier injury depending on IL-22 expression. Collectively, this study probed into the potential molecular mechanism regarding the protective effect of LGG on ALD using animal experiments, providing a potential basis for the treatment of chronic plus binge ALD in clinical practice.

## Materials and methods

### Wild-type mouse models of chronic plus binge ALD and LGG experiment

The present study used 8- to 10-week-old male C57BL/6 J mice to construct chronic plus binge ALD model. All animals were acquired from Beijing Vital River Laboratory Animal Technology Co., Ltd (Beijing, China) and received humane care. The animal experiments were performed in accordance with the protocols approved by the Institutional Animal Care and Use Committee of Nanfang Hospital (No. G202010235).

All mice were placed in an environmentally controlled room (temperature: 23°C ± 1°C, humidity: 55% ± 5%, 12-h light/12-h dark, light cycle beginning at 07:00) with unrestricted access to water and food. The C57BL/6 J mice were subjected to a chronic plus a single binge ethanol feeding protocol proposed by the National Institute on Alcohol Abuse and Alcoholism [17]. In brief, these mice were first given the Lieber-DeCarli liquid control diet (F1259SP, Bioserv, Flemington, NJ, USA) for 5 days and further pair-fed with the Lieber-DeCarli liquid control or ethanol diet (F1258SP, Bioserv, Flemington, NJ) for 10 days. At day 11, the ethanol-treated mice were subjected to 5 g/kg ethanol (140,029, JiuYi Reagent Co., Ltd., Nanjing, Jiangsu, China) while control-treated mice were given 9 g/kg maltose dextran (00895, Sigma-Aldrich, St. Louis, MO, USA).

For LGG treatment, mice received live LGG (suspended in physiological saline, 53,103, American Type Culture Collection, Manassas, VA, USA) at a dose of 10^9^ colony-forming units (CFU)/day for 15 days by gavage [18]. The control samples were fed with the same volume of physiological saline (PB180353, Procell, Wuhan, Hubei, China).

For IL-22 knockdown experiments, IL-22 adenoviral vectors (Ad-shRNA-IL-22) were constructed under the AdMax system (Hanbio Biotechnology Co., Ltd., Shanghai, China) and a negative control (Ad-shNC, Hanbio Biotechnology, Shanghai, China) was served as the control. One dose of Ad-shRNA-negative control (shNC, 1 × 10^9^ PFU/mouse, intravenous injection (i.v.)) and Ad-shRNA-IL-22 (1 × 10^9^ PFU/mouse, i.v.) was given on the day prior to ethanol feeding.

RETRACTED

On the last day of feeding, after gavage for 8 hours (h), mice were euthanized by a continuous exposure to 5% isoflurane (Keyuan Pharma, Jinan, Shandong, China) until 1 min after the breath stop according to the 2013 American Veterinary Medical Association Guidelines for the Euthanasia of Animals. Then, blood, liver, and colon tissues from mice were collected.

### RNA isolation and quantitative real-time polymerase chain reaction (qRT‐PCR)

RNA samples were isolated using TRIzol reagent (15596018, Invitrogen, Carlsbad, CA, USA) following the instructions, and then reverse-transcribed to cDNA by the SuperScript IV Reverse Transcript (18090200, Thermo Fisher Scientific, Waltham, MA, USA). Next, quantitative PCR was carried out via PowerUp™ SYBR™ Green Master Mix (A46113, Thermo Fisher Scientific) in a 96-well PCR plate on the 7500 Sequence Detection system (4351107, Applied Biosystems, Foster City, CA, USA). The 2^–ΔΔCT^ method was utilized to calculate the relative mRNA expression using β-actin as an internal reference [19]. The primer sequences were as follows: IL-22 forward, 5'-GTCAACCGCACCTTTATGCT-3', reverse, 5'-CCCCGATGAGCCGGACA-3'; and β-actin forward, 5'-GCGGGCGACGATGCT-3', reverse, 5'-GCCACAGGATTCCATACCCA-3'.

### Enzyme-linked immunosorbent assay (ELISA)

IL-22 level was determined with an ELISA kit (PI591, Beyotime, Jiangsu, China) based on the manufacturer’s protocol. Briefly, each well of enzyme-labeled-coated plate was added with 40 μl of sample analysis buffer followed by the addition of 40 μl sample and 100 μl of enzyme-labeled reagent in turn. After cultivation with biotinylated antibodies, streptavidin-conjugated horseradish peroxidase (HRP) was added into each well and reacted with HRP substrate solution. The plates were read at a wavelength of 450 nm using a Multiskan FC device (1410101, Thermo Fisher Scientific).

### Assessment of liver injury

Blood was collected and serum was separated through centrifugation at 4000 rpm at 4°C for 10 minutes (min). The levels of alanine aminotransferase (ALT), triglyceride (TG), and aspartate aminotransferase (AST) in serum were detected utilizing the reagent kits as per the manufacturer’s specification. ALT reagent (C009-1-1), TG (A110-1-1), and AST (C010-1-1) were obtained from Nanjing Jiancheng Bioengineering Institute (Nanjing, Jiangsu, China).

To measure the levels of ALT and AST, the matrix solution was pre-heated in a 37°C thermostat, 20 μl of which was added to the 96-well plate. Next, 5 μl of serum samples were introduced into the assay well which was then placed in the 37°C thermostat for 30 min. Subsequently, 2,4-dinitrophenylhydrazine solution was used to stop the reaction. 20 min later, sodium hydroxide solution was supplied to each well for color development. Next, the absorbance was measured at 505 nm using the Multiskan FC device (1410101, Thermo Fisher Scientific).

RETRACTED

For hepatic TG analysis, liver samples were homogenized in ice-cold phosphatic buffer solution. The supernatant solution was obtained by centrifuging (12,000 *g*) at 4°C for 10 min. 2.5 μl of samples were mixed with 250 μl working solution. After incubation for 10 min, the absorbance was measured at 510 nm through the Multiskan FC device (1410101, Thermo Fisher Scientific).

### Hematoxylin eosin (HE) staining

The liver and colon tissues were fixed in 4% paraformaldehyde (C104190, Aladdin, Shanghai, China), embedded in paraffin (P100933, Aladdin), and sliced into 5-µm-thick sections. After a day of baking at 37°C, these sections were immersed in xylene (X139941, Aladdin) twice for 10 min, 100% ethanol (140,029, JiuYi Reagent Co., Ltd) for 5 min, 80% ethanol for 5 min, and 70% ethanol for 5 min. Upon rinsing with tap water, these sections were stained with hematoxylin (H292717, Aladdin) for 5 min, and then soaked in tap water for 15 min. Afterward, the sections were subjected to 70% ethanol for 5 min and 80% ethanol for 5 min, then stained with eosin (E301878, Aladdin) for 1 min, and sealed with neutral resin (N305043, Aladdin). Finally, an inverted microscope (XSP-8CA, Shanghai Optical Instrument Factory, Shanghai, China) was served to observe and photograph the pathological changes.

### Western blot

Protein samples were harvested from the colon tissues by Radio Immunoprecipitation Assay Lysis Buffer (P0013B, Beyotime) containing protease inhibitors. A bicinchoninic acid protein assay kit (ab102536, Abcam, Cambridge, MA, USA) was utilized to determine the protein concentration. Equal amounts of proteins were subjected to 10% sodium dodecyl sulfate-polyacrylamide gel electrophoresis (SDS-PAGE, P0670, Beyotime) prior to being transferred onto polyvinylidene fluoride (PVDF, FFP24) membranes, which were then blocked by 5% skim milk. Thereafter, these membranes were incubated with primary antibodies at 4°C for 24 h, including anti-tight junction protein 1 (ZO-1, 1/1000, ab216880, Abcam), anti-Claudin-1 (1/2000, ab180158, Abcam) and anti-β-actin (1 µg/ml, ab8226, Abcam) antibodies. Subsequently, these membranes underwent 1-h cultivation with HRP-conjugated goat anti-rabbit secondary antibody (1/2000, ab6721, Abcam) or goat anti-mouse secondary antibody (1/2000, ab205719, Abcam) for visualization. β-actin was regarded as an internal reference. The protein band was obtained by an enhanced chemiluminescence detection system (Amersham Biosciences, Piscataway, NJ, USA).

RETRACTED

### Statistical analysis

All statistical analyses were conducted using GraphPad Prism 8.0 software (San Diego CA, USA) and the data were expressed as mean ± standard deviation. One-way analysis of variance was adopted to compare the differences among four groups, together with a Bonferroni *post hoc* test. The *p* value less than 0.05 was perceived as statistical significance.

## Results

In this study, we surmised that LGG may effectively ameliorate alcohol-induced liver injury through regulating the IL-22 signaling pathway. Wild-type mouse model of chronic plus binge ALD was established to explore the effect of LGG on the expression level of IL-22, liver injury and intestinal barrier. This study dug deeply into the potential molecular mechanism concerning the protective effect of LGG on ALD using animal experiments. The results indicated that LGG alleviated alcohol-induced liver and intestinal barrier injury by modulating IL-22 expression, providing a potential basis for the treatment of chronic plus binge ALD in clinical practice.

### LGG affected the expression of IL-22 in the chronic plus binge ALD model

Initially, we constructed a chronic plus binge ALD model to assess the effect of LGG on the level of IL-22 and liver function. As shown in Figure 1(a,b), qRT-PCR and ELISA results revealed that compared with the control, IL-22 level was notably reduced in the model (*p* < 0.01), whereas LGG could rescue such reduction (*p* < 0.01) and dramatically enhanced IL-22 level (*p* < 0.01, Figure 1(a,b)). All these data signified that LGG increased the level of IL-22 in the chronic plus binge ALD model.

**Figure 1.** LGG elevated IL-22 expression and affected alcohol-induced liver functions. (a) The mRNA expression of IL-22 of liver tissues was evaluated by qRT-PCR in control, model, model+LGG, and LGG groups. The 8- to 10-week-old C57BL/6 J mice were used to construct chronic plus binge alcoholic liver disease model. For LGG treatment, mice received live LGG by gavage at a dose of 10^9^ colony-forming units every day for 15 days. The control mice were fed with the same volume of physiological saline. (b) The level of IL-22 in serum was detected by ELISA. (c-e) Levels of ALT (c), AST (d), and TG (e) in serum of mice with different treatments. **p < 0.01, ***p < 0.001 vs. Control; ^^^*p* < 0.05, ^^^^*p* < 0.01, ^^^^^*p* < 0.001 vs. model; ^#^*p* < 0.05, ^##^*p* < 0.01, ^###^*p* < 0.001 vs. model+LGG. LGG, *Lactobacillus rhamnosus* GG; IL-22, interleukin 22; qRT-PCR, quantitative real-time polymerase chain reaction; ELISA, enzyme-linked immunosorbent assay; ALT, alanine aminotransferase; TG, triglyceride; AST, aspartate aminotransferase.

RETRACTED

### LGG improved liver injury in the chronic plus binge ALD model

We detected the levels of ALT, TG, and AST to evaluate the effect of LGG on liver function. Results exhibited in Figure 1(c-e) demonstrated that these levels were notably elevated in the chronic plus binge ALD model by contrast with those in the control (*p* < 0.001), while such elevation can be offset by introduction of LGG (*p* < 0.05). Additionally, compared with LGG treatment in the model, LGG treatment under the basic condition could significantly reduce the levels of ALT and AST (*p* < 0.05, Figure 1(c-e)).

Moreover, we evaluated the effect of LGG on the histopathological morphology of liver in mouse model through HE staining, and unveiled that alcohol treatment resulted in liver injury, inflammatory infiltration, steatosis, and lipid droplets elevated (Figure 2(a)). Fortunately, LGG could reduced this liver injury, steatosis, and lipid droplets in the model (Figure 2(a)). Collectively, all these findings illustrated that LGG might play a protective role in the alcohol-damaged liver tissues.

**Figure 2.** LGG alleviated injury of liver and intestinal barrier caused by alcohol. (a) Representative HE staining of liver tissues in different treatments, alcohol treatment resulted in liver injury, inflammatory infiltration, steatosis and lipid droplets elevated, while LGG could reduced this liver injury. Magnification, ×400; Scale bar, 100 μm. (b) Representative HE staining of colon tissues in different treatments. Magnification, ×40; Scale bar, 100 μm. (c-d) Protein levels of ZO-1 and Claudin-1 in colon tissues were determined by western blot analysis. (c) Representative protein bands. (d) Quantification of proteins. The 8- to 10-week-old C57BL/6 J mice were used to construct a chronic plus binge alcoholic liver disease model. For LGG treatment, mice received live LGG by gavage at a dose of 10^9^ colony-forming units every day for 15 days. The control mice were fed with the same volume of physiological saline. ***p < 0.01 vs. Control; ^^^p < 0.05, ^^^^p < 0.01 vs. model; ^##^p < 0.01 vs. model+LGG. LGG, *Lactobacillus rhamnosus* GG; HE, hematoxylin eosin; ZO-1, tight junction protein 1.

### LGG alleviated intestinal barrier injury caused by alcohol

The effect of LGG on the colon tissues in alcohol-exposed mice was evaluated via HE staining. Compared with the control, the model mice showed severe injury in intestinal barrier, intestinal villi become thinner, shorter and irregular, which could be prominently alleviated after receiving gavage administration with LGG (Figure 2(b)).

RETRACTED

Zonula occluden-1 (ZO-1) and Claudin-1 are instrumental in mediating tight junction barrier function, and also the main functional regulatory factors of tight junction [20]. Therefore, we investigated the impact of LGG on protein levels of ZO-1 and Claudin-1 in the colon using western blot analysis. The data demonstrated that protein levels of ZO-1 and Claudin-1 were both markedly lessened in the model group (*p* < 0.001, Figure 2(c,d)), but, comparatively, was signally augmented in the model+LGG group, and most augmented in the LGG group (*p* < 0.05, Figure 2(c,d)). All these discoveries manifested that gavage administration with LGG could alleviate intestinal barrier injury in mice with chronic plus binge ALD.

### The amelioration of alcohol-induced liver injury by LGG was dependent on IL-22 expression

Since our previous results proved that LGG regulated IL-22 expression as well as ameliorated liver injury in the chronic plus binge ALD model, we wondered whether the amelioration of alcohol-induced liver injury by LGG was associated with IL-22 expression. As shown in Figure 3(a), the mRNA level of IL-22 in liver tissues was significantly reduced in shIL-22 group than that in shNC group (*p* < 0.001, Figure 3(a)). Also, the mRNA level of IL-22 was dwindled in the model+LGG+shIL-22 group compared with model+LGG+shNC group (*p* < 0.001, Figure 3(a)). Moreover, we observed that compared with shNC group, the levels of ALT, TG, and AST in serum were promoted in shIL-22 group (*p* < 0.05, Figure 3(b-d)). As expected, levels of these three factors were increased in the model+LGG+shIL-22 group as comparison with those in the model+LGG+shNC group (*p* < 0.05, Figure 3(b-d)).

**Figure 3.** LGG affected alcohol-induced liver damage by regulating IL-22 expression. (a) The mRNA expression of IL-22 in liver tissues was detected by qRT-PCR after downregulation of IL-22. (b-d) Levels of ALT (b), AST (c), and TG (d) in serum of mice with different treatments. The 8- to 10-week-old C57BL/6 J mice were used to construct a chronic plus binge alcoholic liver disease model. For LGG treatment, mice received live LGG by gavage at a dose of 10^9^ colony-forming units every day for 15 days. One dose of Ad-shRNA-NC (shNC, 1 × 10^9^ PFU/mouse, i.v.) and Ad-shRNA-IL-22 (1 × 10^9^ PFU/mouse, i.v.) was given on the day prior to ethanol feeding. *p < 0.05, **p < 0.01, ***p < 0.001 vs. model+LGG+shNC; ^&^*p* < 0.05, ^&&^*p* < 0.01, ^&&&^*p* < 0.001 vs. shNC. LGG, *Lactobacillus rhamnosus* GG; IL-22, interleukin 22; qRT‐PCR, quantitative real-time polymerase chain reaction; ALT, alanine aminotransferase; TG, triglyceride; AST, aspartate aminotransferase; NC, negative control, Ad, adenoviral vector.

RETRACTED

In addition, we noticed that shIL-22 group presented damaged liver, steatosis, and lipid droplets compared with shNC group (Figure 4(a)), and the condition was aggravated in model+LGG+shIL-22 group by comparison with that in model+LGG+shNC group (Figure 4(a)). Together, these findings implied that the amelioration of alcohol-induced liver injury by LGG depended on IL-22 expression.

**Figure 4.** LGG alleviated alcohol-induced injury of liver and intestinal barrier through regulation of IL-22 expression. (a) Representative HE staining of liver tissues in different treatments. Magnification, ×400; Scale bar, 100 μm. (b) Representative HE staining of colon tissues in different treatments. Magnification, ×40; Scale bar, 100 μm. (c-d) Protein levels of ZO-1 and Claudin-1 in colon tissues were determined by western blot analysis. (c) Representative protein bands. (d) Quantification of proteins. The 8- to 10-week-old C57BL/6 J mice were used to construct a chronic plus binge alcoholic liver disease model. For LGG treatment, mice received live LGG by gavage at a dose of 10^9^ colony-forming units every day for 15 days. One dose of Ad-shRNA-NC (shNC, 1 × 10^9^ PFU/mouse, i.v.) and Ad-shRNA-IL-22 (1 × 10^9^ PFU/mouse, i.v.) was given on the day prior to ethanol feeding. **p < 0.01, ***p < 0.001 vs. model+LGG+shNC; ^&&^*p* < 0.01, ^&&&^*p* < 0.001 vs. shNC. LGG, *Lactobacillus rhamnosus* GG; HE, hematoxylin eosin; ZO-1, tight junction protein 1.

### The amelioration of alcohol-induced intestinal barrier damage by LGG was dependent on IL-22 expression

Given that the amelioration of the alcohol-induced intestinal barrier damage by LGG treatment might be associated with IL-22 expression, we examined the effect of IL-22 silencing on the intestinal barrier injury and protein expressions of ZO-1 and Claudin-1 through HE staining and western blot, respectively. In light of Figure 4(b), intestinal barrier injury was severer in the shIL-22 group than in shNC group. Similarly, intestinal barrier dysfunction, intestinal villi become thinner, shorter and irregular, was exacerbated in model+LGG+shIL-22 group (Figure 4(b)). Meanwhile, the western blot analysis revealed that expression levels of ZO-1 and Claudin-1 were both downregulated in shIL-22 group when compared to those in the shNC group (*p* < 0.01, Figure 4(c,d)), and were also inhibited in model+LGG+shIL-22 group by contrast with those in model+LGG+shNC group (*p* < 0.01, Figure 4(c,d)). Taken together, these data manifested that the amelioration of alcohol-induced intestinal barrier damage by LGG also relied on IL-22 expression.

RETRACTED

## Discussion

In the present study, we constructed an alcohol-induced ALD model to evaluate the potential mechanism concerning the effect of LGG on the intestinal barrier and liver injury. The results uncovered that supplementation of LGG could significantly ameliorate the liver function damage caused by long-term alcohol feeding. Moreover, the protective effect of LGG was associated with the IL-22 signaling pathway. LGG played its hepatoprotective activity by upregulating the expressions of IL-22 and intestinal barrier-related proteins. These data implicated that the IL-22 signaling pathway acts a crucial role in the probiotics LGG treatment of ALD.

Our results verified previous reports that probiotics ameliorate liver injury caused by chronic alcohol and the integrity of intestinal epithelial cell barrier function is a potential mechanism of liver injury [21,22]. Forsyth et al. reported that probiotics LGG could effectively reduce the alcohol-induced oxidative stress to maintain the intestinal barrier function and thus improve the liver injury using an animal model of ALD [23]. Probiotics also prevented liver damage in acute alcohol-fed models [24]. In this study, a model of chronic plus binge ALD was established. The data revealed that supplementation with LGG to model mice diminished the levels of ALT, TG, and AST. The following HE staining analysis confirmed that LGG reversed liver damage and steatosis induced by alcohol, which were consistent with previous studies.

Previous studies pointed out that, in a mouse model of ALD, chronic alcohol brings about loss of intestinal tight junctions and increased intestinal permeability [25,26]. Indeed, it has been revealed that LGG effectively protects intestinal barrier function [27,28]. LGG treatment protects intestinal epithelial cells from oxidant stress, possibly by maintaining cytoskeletal integrity [29]. Short-term oral supplementation of certain probiotics is more effective than standard treatment alone in promoting the recovery of intestinal flora and improving alcohol-caused liver injury [30]. As early as 1993, it has been confirmed that LGG alleviated the increase in intestinal mucosal permeability induced by milk in suckling mice [31]. In this study, LGG was confirmed to mitigate intestinal barrier damage by HE staining analysis, which well supported the results of previous studies. Additionally, the disintegration of tight junction proteins was found to be a contributing factor in the pathogenesis of chronic alcohol-caused intestinal barrier dysfunction [25]. In this study, ALD induction was associated with downregulations of ZO-1 and Claudin-1 in colon tissues. However, LGG effectively inhibited ALD-related decreases in the expression levels of these intestinal barrier-related proteins. Combined with our results and previous reports, we can conclude that LGG improves intestinal barrier function and ameliorate alcohol-caused liver injury.

RETRACTED

Currently, the action mechanism of LGG in protecting against intestinal barrier and alcoholic liver injury is still unclear. As we know, probiotics could alter the gut microbiota in such a way that the intestinal cavity is altered in favor of the anti-inflammatory environment, thereby reducing the production of pro-inflammatory bacterial products and improving barrier integrity [23]. This reminded us to think about whether or not the inflammatory pathway is involved in the hepatoprotective effect or the restoration effect of intestinal barrier function of LGG in alcohol-induced mice. In the intestine, IL-22 was discovered to support the regeneration of intestinal epithelial barrier functions [32]. Moreover, IL-22 is implicated in several aspects of intestinal epithelial barrier functions, including epithelial cell growth and permeability, mucus and antimicrobial protein production, and complement production [33]. In our initial experiments, we observed that IL-22 expression was obviously upregulated after LGG treatment in chronic plus binge ALD mouse models, hinting that IL-22 may be involved in the protective role of LGG in intestinal barrier. As expected, downregulation of IL-22 aggravated liver function and intestinal barrier, suggesting that LGG prevented chronic alcohol-induced intestinal barrier and liver injury partly via regulating the expression of IL-22, which may be the potential mechanism of its beneficial action.

## Conclusion

In summary, this study corroborates that LGG treatment in chronic plus binge ALD mouse model protects against alcohol-induced intestinal barrier and liver injury. Moreover, this is the first report to reveal that IL-22 signaling pathway plays a vital role in the process of LGG protection of ALD. However, a limitation should be addressed here is that this study is only conducted on liver and colon samples from healthy male mice. Further studies should be carried out in females, infant, and aged mouse models. Nevertheless, the present study explores the potential mechanism of the role of LGG in liver protection, providing a theoretical basis for the further optimization of probiotics in the prevention and therapy of ALD.

## Data Availability

The analyzed data sets generated during the study are available from the corresponding authors on reasonable request.
